# The Predictive Efficacy of Serum Exosomal microRNA-122 and microRNA-148a for Hepatocellular Carcinoma Based on Smart Healthcare

**DOI:** 10.1155/2022/5914541

**Published:** 2022-01-04

**Authors:** Peng Deng, Mi Li, Yuni Wu

**Affiliations:** Department of Oncology, Chongqing General Hospital, Chongqing 610095, China

## Abstract

**Objective:**

Hepatocellular carcinoma (HCC) remains a devastating tumor globally. Serum exosomes are reliable biomarkers for tumors, including HCC. Hence, this study explored the efficacy and mechanism of serum exosomes in HCC.

**Methods:**

microRNA (miR)-122 and miR-148a expressions in serum exosomes from HCC patients and healthy subjects and their predictive efficacy for HCC were detected. Correlation between serum exosomal miR-122/148a expressions with survival rate, clinical stage, lymph node metastasis, and tumor differentiation level and levels of HCC-related serum markers (CA199, FucAFP, ALD-A, and AFu) were detected. PAX2 staining intensity and expression in HCC were measured. PAX2 predictive efficacy for HCC and its correlation with clinical stage, lymph node metastasis, tumor differentiation level, and HCC-related serum marker levels were analyzed. The targeted binding relationship between miR-122 and miR-148a and PAX2 was predicted and verified.

**Results:**

Serum exosomal miR-122 and miR-148a expressions were downregulated in HCC, showing potent predictive efficacy for HCC, which was negatively related to clinical stage and lymph node metastasis and positively related to tumor differentiation level, patient survival rate, and HCC-related serum marker levels. PAX2 showed increased staining intensity and expression in HCC, together with high predictive efficacy for HCC. PAX2 expression showed a positive correlation with clinical stage and lymph node metastasis and a negative correlation with tumor differentiation level and HCC-related serum marker levels. miR-122 and miR-148a conjointly targeted PAX2 in HCC.

**Conclusion:**

We demonstrated that serum exosomal miR-122 and miR-148a played a predictive role and were linked to prognosis in HCC via interactions with PAX2.

## 1. Introduction

Hepatocellular carcinoma (HCC), as a frequent malignancy that usually occurs in the presence of chronic liver disease, accounts for 75–85% of primary liver cancers and contributes to the vast majority of cancer-related deaths [1, 2]. HCC develops mostly as a consequence of hepatitis B infection; in addition, other risk factors including genetic causes, excessive drinking, hepatitis C infection, and fatty liver disease also contribute to HCC initiation and progression [3, 4]. Due to insidious symptoms in the early stage and subsequent rapid tumor development, a majority of HCC patients are not diagnosed until the late stage, during which HCC is largely incurable due to the low therapeutic response rate and apparent drug resistance [5, 6]. Surgical resection and liver transplantation are still two standard methods for treating HCC; however, the recurrence rate after radical resection and transplantation remains high, notably reducing the long-term survival of HCC patients [7–9]. Therefore, novel predicative biomarkers are in urgent need for promoting HCC diagnosis as well as improving the prognosis.

Exosomes are characterized by small bilipid protein structures with a diameter of 30–150 nm and show the presence of almost all biological fluids including serum, which makes them recognized as reliable biomarkers for cancer prognosis and diagnosis [10]. Exosomes harbor abundant biological cargoes, such as DNA, microRNAs (miRs), and proteins, which underlie their potential to be biomarkers for diagnostic applications [11]. miRs, defined as a group of small endogenous noncoding RNAs, are potent regulators of posttranscriptional gene expression, promising to be candidates for developing biomarkers [12, 13]. Serum exosomal microRNAs (miRs) are very stable and can act as effective biomarkers for early cancer diagnosis [14]. Accumulating studies have demonstrated that serum exosomal miRs have great value in HCC diagnosis and therapy and can also be used as novel hallmarks for HCC recurrence prediction [6, 15].

Therefore, it was reasonable to hypothesize that serum exosomes may possess an underlying value in HCC prediction and prognosis via carrying miRs through possible mechanisms. Consequently, a series of predictions and experiments were performed to determine the role of HCC-related serum exosomal miRs and their related mechanisms in HCC prediction and prognostic evaluation with the purpose to provide some novel insights for HCC treatment.

## 2. Materials and Methods

### 2.1. Clinical Sample Collection

HCC serum samples were collected from Chongqing General Hospital. HCC patients had no history of acute, chronic, or malignant diseases or surgery in the previous 12 months based on the screening results of the physical examination center of Chongqing General Hospital. Histologically, HCC patients were confirmed with no radiotherapy and chemotherapy history and no acute/chronic inflammation signs. Normal subjects (*n* = 31) were matched with HCC patients (*n* = 59) by age and gender. This study got approval from the Ethics Committee of Chongqing General Hospital. All subjects signed informed consent. All experiments were performed following the guidelines and principles of the Declaration of Helsinki.

Peripheral blood samples were collected in the serum separation tube and treated within 2 h. After centrifugation (1200*g*, 4°C, and 10 min) of the blood samples, the supernatant was absorbed and centrifuged (3,000*g*, 4°C, and 15 min). Next, the supernatant was crushed into several equal parts and stored at −80°C.

### 2.2. Extraction of Serum Exosomes

The exosomes were separated using gradient centrifugation as previously described [16]. Specifically, serum samples were unfrozen on ice. Next, serum (1 mL) was diluted in phosphate-buffered saline (PBS, 11 mL) and then ultracentrifuged (150,000*g*, 4°C overnight). After discarding the supernatant, the precipitate was rinsed with PBS (11 mL), followed by centrifugation (150,000*g*, 4°C, and 2 h). Afterwards, after the supernatant was removed, the precipitate underwent a resuspension in PBS.

### 2.3. Transmission Electron Microscope (TEM) Analysis

Exosome samples were diluted using PBS at an appropriate volume. Next, the diluted exosomes (10 *μ*L) were added to the copper mesh for 1 min with excess liquid absorbed using filter paper, followed by a 1min staining with 2% uranyl acetate (10 *μ*L) with excess staining solution absorbed using filter paper. Next, the copper mesh underwent a 15-minute air-drying and was imaged on an FEI Tecnai G2 Spirit TEM (Thermo Fisher Scientific Inc., Waltham, MA, USA) at a voltage of 120 kV.

### 2.4. Nanoparticle Tracking Analysis (NTA)

NTA was conducted for the determination of exosome size and distribution utilizing the NanoSight NS300 system and NTA 2.3 (Malvern Instruments Ltd., Malvern, UK) in compliance with the instructions of the manufacturer.

### 2.5. Flow Cytometry

Anti-CD63, anti-CD81, and anti-CD47 antibodies or PI were used to label the extracted exosomes. A flow cytometer was used to excitate 525/620 nm band-pass filters at 488 nm wavelength for detecting FITC/PI fluorescence to evaluate the positive rates of CD63, CD81, CD47, and PI in the extracted exosomes.

### 2.6. Detection of HCC-Related Serum Markers

Concentrations of cancer antigen 199 (CA199), fucosylated alpha-fetoprotein (FucAFP), aldolase A (ALD-A), and Alpha-L-fucosidase (AFU) were detected using enzyme-linked immunosorbent assay kits (Nanjing JianCheng Bioengineering Institute, Nanjing, Jiangsu, China). All operations were carried out as per the kit instructions.

### 2.7. Dual-Luciferase Reporter Gene Assay

The binding relationship of miR-122/148a and PAX2 was first predicted through StarBase (https://starbase.sysu.edu.cn/). The wild-type (WT) PAX2 3′UTR fragment containing miR-122/148a binding sites or mutant (MT) (in the absence of predicted miR target sequence) was inserted into pmirGLO (Shanghai Generay Biotech Co., Ltd., Shanghai, China) plasmid. The reporter plasmid (pmirGLO-PAX2-WT/MT) was cotransfected with miR-122/148a mimic or mimic NC into HEK293T cells. After 48 h of transfection, cell lysate was collected and luciferase activity was measured using Tecan Infinite M200 PRO instrument and Dual-Luciferase Reporter System (Promega Corp., Madison, Wisconsin, USA). The firefly luciferase fluorescence intensity was standardized using Renilla luciferase fluorescence intensity.

### 2.8. Bioinformatics Analysis

HCCGSE104251 and GSE138178 microarrays were obtained from the Gene Expression Omnibus (GEO) database (https://www.ncbi.nlm.nih.gov/geo/), which were then normalized using the R language limma package (https://cran.r-project.org/web/packages/pheatmap/) with |logFC| > 2 and adj. *p* < 0.05 as the screening thresholds. The heatmaps were drawn. The targeted binding relationship between miR-122/148a and PAX2 was predicted through StarBase (https://starbase.sysu.edu.cn/). The relationship between miR-122 and miR-148a expressions and the survival rate of HCC patients was measured using the KM-Plotter website (https://kmplot.com/analysis/). The staining intensity of paired box (PAX) 2, cyclinD1 (CCND1), myelocytomatosis viral oncogene homolog (MYC), neural precursor cell expressed, developmentally downregulated 4 (NEDD4), and C-X-C motif chemokine ligand 5 (CXCL5) in normal liver tissues and HCC tissues was determined through the Human Protein Atlas website (https://www.proteinatlas.org/).

### 2.9. Reverse Transcription-Quantitative Polymerase Chain Reaction (RT-qPCR)

cDNA synthesis was performed using the All-in-One™ miRNAFirst-Strand cDNA Synthesis Kit (GeneCopoeia, Rockville, MD, USA) as per the manufacturer's protocols. Reverse transcription was accomplished via a 60-minute incubation of the mixture at 37°C and then a 5-minute incubation at 85°C, followed by storage at 4°C. RT-qPCR was carried out utilizing ChamQ SYBR qPCR Master Mix (NanJing Vazyme Biotech Co., Ltd, Nanjing, Jiangsu, China) as per the instructions of the manufacturer. All reactions were checked three times. miRprimer2 software 32 was used for miRNA forward primer design, and its synthesis was finished by Nanjing Genscript Technology Co., Ltd. (Nanjing, Jiangsu, China). RT-qPCR was carried out on the StepOnePlus real-time PCR system (Applied Biosystems, Waltham, MA, USA) under the conditions of 3 min at 95°C, and then 40 cycles of 10 s at 95°C and 30 s at 60°C. The geometric mean of the internal reference was used for RT-qPCR value normalization, and the relative expression was determined using the 2^−ΔΔCt^ method.

### 2.10. Statistical Analysis

SPSS 21.0 (IBM Corp., Armonk, NY, USA) was utilized to analyze data. The Kolmogorov–Smirnov test confirmed that data were normally distributed. The results were represented as mean ± standard deviation. The comparison between the two groups was analyzed using a *t*-test. A comparison among multiple groups was analyzed using one-way and two-way analysis of variance (ANOVA) followed by Tukey's multiple comparison test. Fisher's exact test was utilized for measurement data. Correlation was analyzed utilizing Pearson's correlation coefficient test, and a receiver operating characteristic (ROC) curve was drawn to evaluate the predictive efficacy of miR-122/148a and PAX2 for HCC. The *p* value was gained from a two-sided test. *p* < 0.05 meant statistically significant.

## 3. Results

### 3.1. Serum Exosomes in HCC Patients Were Successfully Extracted

First, exosomes were extracted from the serum of 31 healthy subjects and 59 HCC patients using gradient centrifugation. The size of the extracted particles was analyzed using the NanoSight NS300 system and NTA 2.3 software, which was observed to be about 92.46 ± 2.41 nm (Figure 1(a)). In addition, the extracted particles were found to be barrel-shaped, ellipsoidal, or round, with a diameter of about 100 nm under a TEM (Figure 1(b)). To further exclude the influence of apoptotic bodies on the subsequent experimental results, we used PI staining and observed that the extracted exosomes were negative for PI staining, as shown by flow cytometry results (Figure 1(c)). Exosome specific surface markers (CD63, CD81, and CD47) were further determined using flow cytometry, and it was found that CD63, CD81, and CD47 showed positive expression in the extracted exosomes (Figure 1(d)). From all the abovementioned, we confirmed that the extracted particles were in line with the characteristics of exosomes.

### 3.2. miR-122/148a Was Poorly Expressed in HCC Patient Serum Exosomes and Correlated with Prognosis

Firstly, differentially expressed miRs in serum exosomes of 5 HCC patients and 5 healthy subjects in the GSE104251 dataset from the GEO database (https://www.ncbi.nlm.nih.gov/geo/) were analyzed, and 179 differentially expressed miRs were screened (Figure 2(a)) based on the threshold of |logFC| > 2 and *p* < 0.05. The first 50 miRs with differential expression were displayed on the heatmap (Figure 2(b)). Next, expressions of the first 6 differentially expressed miRs (miR-122, miR-239, miR-148a, miR-447, miR-681, and miR-581) in serum exosomes of 31 healthy subjects and 59 HCC patients were detected using RT-qPCR. miR-122 and miR-148a were found to be dramatically downregulated in serum exosomes of HCC patients (Figure 2(c)). Meanwhile, the predictive efficacy of the first 6 differentially expressed miRs (miR-122, miR-239, miR-148a, miR-447, miR-681, and miR-581) for HCC patients was measured using an ROC curve. miR-122 and miR-148a showed the largest area under the curve (Figure 2(d)). Subsequently, miR-122 and miR-148 effects on HCC patient survival rate were predicted through the KM-Plotter website (https://kmplot.com/analysis/), and it was found that HCC patients with low expression of miR-122/148a had a lower survival rate (Figure 2(e)). In addition, according to our findings, miR-122/148a expression was negatively correlated with the clinical stage and lymph node metastasis of HCC patients, while positively correlated with the tumor differentiation level (Figures 2(f)–2(h)).

### 3.3. miR-122/148a Expression Was Negatively Correlated with HCC-Related Serum Marker Levels

To further determine the role of miR-122/148a in HCC patients, we further analyzed the relationship between miR-122/148a expression in serum exosomes and the concentration of HCC-related serum markers (CA199, FucAFP, ALD-A, and AFu) in HCC patients. First, levels of CA199, FucAFP, ALD-A, and AFu in 59 HCC patients were found to show an obvious elevation relative to those in 31 healthy subjects (Figures 3(a)–3(d)). Next, as shown by our results, miR-122/148a expression was negatively related to HCC-associated serum marker concentrations (Figures 3(e)–3(h)).

### 3.4. PAX2 Was Highly Expressed in Serum of HCC Patients

Subsequently, we downloaded the HCC GSE138178 microarray (including HCC tissues and normal adjacent liver tissues of 49 HCC patients) from the GEO database (https://www.ncbi.nlm.nih.gov/geo/). By setting the threshold |logFC| >2 and *p* < 0.05, 539 differentially expressed genes were identified (Figure 4(a)). The first 50 differentially expressed mRNAs were displayed in the heatmap (Figure 4(b)). The staining intensity of PAX2, CCND1, MYC, NEDD4, and CXCL5 in normal liver tissues and HCC tissues was further determined through the Human Protein Atlas website (https://www.proteinatlas.org/), which was found to show a notable elevation in HCC tissues compared to that in normal liver tissues (Figures 4(c)–4(g)). Furthermore, PAX2, CCND1, MYC, NEDD4, and CXCL5 expressions in the serum of 31 healthy subjects and 59 HCC patients were detected using RT-qPCR, and they were found to be noticeably increased in the serum of HCC patients relative to those in normal subjects, among which PAX2 exhibited the most significant expression difference (Figure 4(h)).

### 3.5. PAX2 Expression Was Related to HCC Patient Prognosis

To further explore PAX2's role in HCC and its clinical-predictive efficacy, we first used a ROC curve to predict the predictive efficacy of PAX2, CCND1, MYC, NEDD4, and CXCL5 expressions for HCC. PAX2 showed the highest predictive efficacy for HCC (Figure 5(a)). The relationship between PAX2 expression and the clinical stage, lymph node metastasis, and tumor differentiation level of HCC patients was further analyzed. As shown by our results, PAX2 expression showed a positive correlation with clinical stage and lymph node metastasis, while a negative correlation with tumor differentiation level (Figures 5(b)–5(d)). Furthermore, levels of CA199, FucAFP, ALD-A, and AFu were found to be positively correlated with PAX2expression in the 59 HCC patients (Figures 5(e)–5(h)). From all of the abovementioned, PAX2 was crucial in the HCC occurrence and prediction.

### 3.6. miR-122 and miR-148a Conjointly Targeted PAX2

To further determine the regulatory mechanism of miR-122 and miR-148a in PAX2, we first predicted the targeted binding relationship between miR-122/148a and PAX2 via the StarBase website (https://starbase.sysu.edu.cn/), and it was observed that miR-122 and miR-148a could target PAX2 3′UTR sequence (Figures 6(a) and 6(b)). The dual-luciferase reporter gene assay was designed to further verify the above binding relationship. 293 T cells cotransfected with miR-122/148a mimic and PAX2-WT showed remarkably decreased luciferase activity, while those cotransfected with mimic NC and PAX2-MT exhibited no obvious change (Figures 6(c) and 6(d)). Subsequently, we verified that miR-122/148a expression showed a negative correlation with PAX2expression in HCC (Figures 6(e) and 6(f)).

## 4. Discussion

Globally, HCC still accounts largely for tumor-related death [17]. Exosomes, widely distributed in biological fluids including serum, are found to be implicated in tumors via carrying their functional cargos, including miRs, thereby showing potential applications in the therapeutic interventions of tumors [18]. In the present study, we demonstrated that HCC patient serum exosomal miR-122 and miR-148a were predictive factors for HCC and related to HCC patient prognosis, which were mediated by their conjointly targeted PAX2 in HCC.

Serum exosomal miRs promise to be biomarkers for HCC prediction [6, 15]. In addition, as has been reported previously, miR-122 is abundant in the liver, and its reduction plays a pathogenic role in liver diseases [19]. Aberrantly decreased miR-148a expression has been described in multiple tumors, with its depletion frequently related to an advanced clinical stage and metastasis, as well as poor clinical outcome [20]. In the present study, differentially expressed miRs in serum exosomes of HCC patients and healthy subjects were first obtained using the GSE104251 microarray, and then we identified the first 6 differentially expressed miRs, among which miR-122 and miR-148a were the two most downregulated miRs in serum exosomes of HCC patients and showed potent predictive efficacy for HCC, and their expressions were negatively related to the clinical stage and lymph node metastasis, and positively correlated with the survival rate and the tumor differentiation level of HCC patients. Likewise, serum exosomal miR-122 shows an obvious downregulation in HCC patients, promising to be a reliable serological biomarker for HCC [21]. miR-122 expression is tightly linked to tumor size and tumor stage in HCC, and reduced miR-122 expression is associated with the short survival of HCC patients [22]. Numerous studies have demonstrated the abnormally reduced miR-148a expression in HCC [23, 24]. A previous work further pointed out that serum miR-148a expression strongly exhibits a negative correlation with tumor size and tumor-node-metastasis stage in HCC and a positive correlation with overall survival and prognosis of HCC patients [25].

As has been demonstrated previously, FucAFP, AFU, CA199, and ALD-A are effective HCC-specific indexes with their high levels correlated with a high risk of HCC [26–29]. According to our findings, levels of HCC-related serum markers (CA199, FucAFP, ALD-A, and AFu) were obviously elevated in HCC patients, and miR-122/148a expression showed a negative correlation with levels of these indexes. Consistently, downregulated miR-122 has been pointed out to be related to the deregulation of ALD-A in liver disease [30]. miR-122 is negatively linked to AFP, an independent risk factor, in HCC [31].

On the other hand, growing studies have shown that PAX2 acts as an oncogenic gene in diverse cancers, such as endometrial cancer and ovarian cancer [32, 33]. Differentially expressed genes in HCC were screened in this study, and we identified PAX2 as the most remarkably upregulated gene in HCC. In agreement with our observations, in prior work, PAX2 is found dramatically elevated in HCC [34]. PAX2 is proposed to possess a clinical-predictive role in endometrial endometrioid carcinoma [35]. As shown by our results, PAX2 showed strong predictive efficacy for HCC, with its expression positively correlated with clinical stage, lymph node metastasis, and HCC-related serum markers (CA199, FucAFP, ALD-A, and AFu), and negatively correlated with tumor differentiation level. Likewise, it has been shown that upregulated PAX2 is tightly related to HCC cell propagation [36].

To further determine the regulatory mechanism of miR-122/148a in PAX2, we first predicted and then verified that miR-122 and miR-148a conjointly targeted PAX2 in HCC. Consistently, previous work has proposed that PAX2 functions as a serum exosomal miR-targeted gene in HCC [36]. miR-122 exhibits a negative correlation with PAX8 in H9C2 myocytes [37]. Nevertheless, little could be retrieved about PAX2's predictive efficacy in HCC and the interplay between miR-122/148a and PAX2 in HCC, which, on the other hand, demonstrated the novelty of this study.

## 5. Conclusion

All in all, this study supported that HCC patient serum exosomal miR-122 and miR-148a played predictive roles in HCC and were linked to patient prognosis via interactions with their conjointly targeted PAX2 in HCC. miR-122 seemed to have higher relevance to PAX2 expression than miR-148; however, more studies are required to draw a certain conclusion that miR-122 had a more important effect than miR-148. We would like to focus on this issue in our future studies, and we would like to investigate the involvement of other potential targets such as CCND1, MYC, NEDD4, and CXCL5 in the near future. Anyway, these results discovered a novel serum exosome-based therapy for HCC patients and provided therapeutic values for HCC treatment.

## Figures and Tables

**Figure 1:** Serum exosomes in HCC patients are successfully extracted. (a) The size and distribution of exosomes was analyzed using NanoSight NS300 system and NTA 2.3 software; (b) the shape and size of exosomes were detected using a TEM; (c) the positive rate of exosomes was detected by PI staining; (d) the surface marker proteins CD63, CD81, and CD47 of exosomes were determined utilizing flow cytometry. All tests were repeated three times.

**Figure 2:** Serum exosomal miR-122 and miR-148a are poorly expressed in HCC and are correlated with prognosis. (a) Volcano plots for the differentially expressed miRs in serum exosome GSE104251 dataset; (b) a heatmap of the top 50 miRs with the highest degree of differential expression in GSE104251 microarray; (c) RT-qPCR was utilized to measure expressions of miR-122, miR-239, miR-148a, miR-447, miR-681, and miR-581 in serum exosomes of 31 healthy subjects and 59 HCC patients; (d) the predictive efficacy of miR-122, miR-239, miR-148a, miR-447, miR-681, and miR-581 for HCC patients was measured using ROC curves; (e) miR-122/148a effects on HCC patient survival rate were predicted using the KM-Plotter website (https://kmplot.com/analysis/); (f–h) the relationships between miR-122/148a expression and the clinical stage, lymph node metastasis, and tumor differentiation level of HCC patients. All experiments were repeated at least three times, and each point represented one subject. Data in panel C were analyzed utilizing the unpaired *t*-test. ^*∗*^*p* < 0.05;  ^*∗∗*^*p* < 0.01;  ^*∗∗∗*^*p* < 0.001.

**Figure 3:** miR-122/148a expression is negatively related to levels of HCC-related serum markers. (a–d) Concentrations of CA199, FucAFP, ALD-A, and AFu in 59 HCC patients were detected; (e–h) the correlation of miR-122/148a expression with the serum levels of CA199, FucAFP, ALD-A, and AFu was analyzed. Data were analyzed using the unpaired *t*-test.  ^*∗∗∗*^*p* < 0.001.

**Figure 4:** PAX2 is highly expressed in serum of HCC patients. (a) Volcano plots for the differentially expressed mRNAs in the GSE138178 dataset; (b) a heatmap of the top 50 differentially expressed mRNAs in the GSE138178 dataset; (c–g) the staining intensities of PAX2, CCND1, MYC, NEDD4, and CXCL5 in normal liver tissues and HCC tissues were determined through the Human Protein Atlas website (https://www.proteinatlas.org/); (h) PAX2, CCND1, MYC, NEDD4, and CXCL5 expressions in the serum of 31 healthy subjects and 59 HCC patients was detected using RT-qPCR. Data in panel H were analyzed utilizing the unpaired *t*-test.  ^*∗∗*^*p* < 0.01;  ^*∗∗∗*^*p* < 0.001.

**Figure 5:** PAX2 expression is related to the prognosis of HCC patients. (a) The ROC curve was used to predict the predictive efficacy of PAX2, CCND1, MYC, NEDD4, and CXCL5 expressions in HCC patients; (b–d) the relationship between PAX2 expression and clinical stage, lymph node metastasis, and tumor differentiation level of HCC patients was analyzed; (e–h) the correlation between levels of CA199, FucAFP, ALD-A, and AFu and PAX2 expression in 59 HCC patients was analyzed. Each experiment was done three times repeatedly.  ^*∗∗*^*p* < 0.01;  ^*∗∗∗*^*p* < 0.001.

**Figure 6:** miR-122 and miR-148a jointly target PAX2. (a, b) The targeting binding sites between miR-122/148a and PAX2 were predicted through the StarBase website (https://starbase.sysu.edu.cn/); (c, d) The dual-luciferase reporter gene assay was designed to further verify the targeted binding relationships between miR-122/148a and PAX2; (e, f) Pearson's correlation coefficient test was used to analyze the correlation between miR-122/148a expression and PAX2 expression. Each experiment was done three times repeatedly.  ^*∗∗*^*p* < 0.01;  ^*∗∗∗*^*p* < 0.001.

## Data Availability

The datasets used and/or analyzed during the current study are available from the corresponding author on reasonable request.
